# A Multimodal Fusion Online Music Education System for Universities

**DOI:** 10.1155/2022/6529110

**Published:** 2022-08-09

**Authors:** Peng Liu, Yixiao Cao, Lei Wang

**Affiliations:** ^1^Music College, Cangzhou Normal University, Cangzhou, Hebei 061000, China; ^2^Art Department, Criminal Investigation Police University of China, Shenyang, Liaoning 110000, China

## Abstract

In the context of Internet technology, the integration of information technology and education is a powerful supplement to the traditional teaching model of higher education. Online learning has become the new development direction of the education industry in the network era. To address the problems of serious difficulty in completing online teaching tasks, difficulty in monitoring teaching effects, and fragmentation of course resources in universities, a multimodal music knowledge graph is constructed. A personalized learning strategy based on users' interest is proposed through the mining of online education data, and a music online education system has been developed on this basis. To improve the recommendation accuracy of the model, an embedding propagation knowledge graph recommendation method based on decay factors is proposed. The model considers the changes in the strength of user interest during the intra- and interlayer propagation of the knowledge graph interest map and focuses on higher-order user potential interest representations for enhancing the semantic relevance of multihop entities. The experimental results show that the proposed model brings a good prediction effect on several benchmark evaluation metrics and outperforms other comparative algorithms regarding recommendation accuracy.

## 1. Introduction

With the promotion of the “Internet+ education” model and the development of artificial intelligence, big data, cloud computing, and other technologies, online music education in colleges and universities, as an important means of education informatization, provides a convenient learning platform for learners beyond the restriction of time and space. And learners can access rich learning resources according to their learning interest and needs [1, 2]. Online education in higher education cannot simply refer to the behavior of teachers in the classroom. Still, it refers to teaching activities that are both efficient and more effective, pursuing teachers and students to obtain the maximum teaching effect with the least possible consumption of time and energy [3–5].

However, current online education platforms in the universities are not perfect in terms of function, focusing only on teachers' design and support for learning content, with relatively little attention and support for students' participatory learning and creative activities. The technical design level is still tainted with the old disease of traditional teaching methods and thinking. The development model is not conducive to the construction of an inquiry-based learning environment. It also has a bad impact on teacher-student interaction and creative talent development [6]. Moreover, students' ability to learn independently online is generally not strong. University students do not perform, and they should in terms of learning interest, learning initiative, teaching participation, and mastery of learning methods [7]. In addition, when many university students choose to study a single course of a particular subject through the online education system, they only focus on the limited learning resources provided on the platform which cannot expand their learning to a deeper level [8]. Therefore, to maximize the value of online education, it is necessary to tap into the interest of online education learners. In addition, it helps the platform provide personalized teaching services to learners by understanding their needs.

Personalized course recommendation for online education platforms is also a hot research issue. Current course recommendations are mainly based on collaborative filtering and data mining methods [9]. The literature [10] uses collaborative filtering methods and association rule analysis comparison based on traditional data mining methods to make course recommendations for learners. Literature [11] uses reinforcement learning methods and Markov decision processes to recommend exercises for learners. The recommendations take into account the smoothing of the difficulty of the exercises, review, and prereading, and the level of learner participation. Literature [12] proposes a neural network-based approach to tracking learners' knowledge levels by providing personalized learning path recommendations for learners. Literature [13] proposes a distributed association rule-based mining algorithm that enables more timely delivery of recommended information and improves the efficiency of course retrieval for users. Literature [14] performs learner browsing log mining based on learners' behavior and interest preferences. Deep learning networks build course recommendation strategies based on the new needs of the mined learners to achieve personalized recommendations for learners. However, collaborative filtering approaches treat the recommendation task as a supervised learning problem. It assumes that each student interaction is an independent instance with accompanying information, ignoring the relationship between the instance and the course. In addition, the approach suffers from data sparsity and cold-start problems due to its failure to extract collaborative signals from collective student behavior and therefore cannot build a recommendation model with good performance. To address the above issues, researchers have considered fusing knowledge graphs into collaborative filtering to improve recommendation effectiveness. Literature [15] constructed a knowledge map for computer networking courses, combined knowledge points and exercises to generate information vectors, and recommended final exercises for learners by analyzing learners' log data and using the similarity between wrong answer practice questions and knowledge points. To be able to recommend content to users more accurately, literature [16] proposed the RippleNet model, which mines users' potential preferences by iterating through the knowledge graph and using their historical interactions as seeds to capture their hierarchical interest in a propagation manner. A new recommendation model was developed in literature [17] by using the TransR algorithm to learn the embedding representation of a knowledge graph. The model uses graph attention networks to recursively propagate embedding representations from the neighbors of nodes for enhancing the embedding representation of nodes. Literature [18] proposes a multimodal visual attribute augmented reinforcement learning model to provide recommendations based on multimodal data sources and demonstrates that fusing multimodal data representations can effectively improve the performance of recommendation systems.

Although several of the above methods can use low-dimensional vectors of users and items for interaction computation, multihop relationship mining is achieved by employing knowledge mapping. However, the wide range of user-item interaction types, in reality, makes the potential semantic information of higher-order interactions may be completely different from the original item representation. Moreover, as the level of propagation increases, the higher-order interaction information becomes more ambiguous. To solve the problems, this paper presents a decay factor-based interlayer interest propagation method based on the knowledge graph recommendation method of embedding propagation. It is used to solve the problem of reduced semantic relevance of knowledge that exists during interlevel propagation by focusing on higher-order user potential interest representations. In addition, to alleviate data noise and degradation problems, a purification network with residual blocks is designed to capture the focus of user interest and improve the accuracy of model recommendations.

The innovations and contributions of this paper are as follows:

1. This model focuses on the strength variation of user interest during intra- and interlayer propagation of the knowledge graph interest map layers and is simulated using decay factors
2. The relevance of multihop entity semantics is improved by enhancing the higher-order user potential interest representation

This paper consists of four main parts: the first part is the introduction, the second part is the methodology, the third part is the result analysis and discussion, and the fourth part is the conclusion.

## 2. Methods

### 2.1. Multimodal Knowledge Mapping for Music

Multimodal knowledge graphs are constructed with multimodal semantic relationships between entities and entities in multiple modalities, which are based on traditional knowledge graphs.  Figure 1 gives an overview of the work involved in building a multimodal knowledge graph, i.e., based on a natural language processing perspective and based on a computer vision perspective. The multimodal knowledge graph construction with NLP is relatively mainstream. Still, it has not yet gotten rid of the reliance on the traditional text knowledge graph. The essence of the work is to complement the knowledge graph and to do the discovery of visual relationships and cross-modal entity links between images. The expansion of image entities and the determination of linking relationships mainly rely on the metadata of multimodal data. The construction of a multimodal knowledge map based on a computer vision perspective is built based on scene mapping generation, bridging visual knowledge with external textual knowledge maps.

A knowledge graph in higher education can accurately characterize the connections between various types of knowledge points and their associated teaching resources and play the role of modeling and managing subject resources. In addition, knowledge graphs in universities can also construct learners' learning information and accurately characterize learners' cognitive state. Combining learning resources and learners' learning information, a college education knowledge graph can generate a variety of intelligent educational applications for learners and promote personalized development.

The music online education knowledge graph is a natural language processing task that fuses information and resources from the music domain to extract music knowledge contained in the metadata, audio, video, images, and text and then structures and semantically represents it according to the online education platform model defined by the music domain ontology. The music knowledge graph correlates entities at all levels of music works, music concepts, music content, music characters, and music resources, supporting unified access to music knowledge and profound knowledge discovery.

This paper constructs a multimodal music knowledge graph for online education in higher education. The information in the graph covers auditory, visual, and textual. The music knowledge comes from various data sources such as audio, sheet music, chants, and metadata. The fused knowledge types include external descriptive information and music content information. It supports knowledge retrieval and knowledge discovery based on music content, as shown in Figure 2.

#### 2.1.1. Music Knowledge Extraction

Knowledge extraction is the process of extracting the knowledge contained in a data source by employing identification, understanding, etc. Music content data is a unique object for knowledge extraction in the music domain. The three main types of music content data, audio, score, and vocals, correspond to different knowledge extraction methods.

*(1) Audio Knowledge Extraction*. Audio knowledge extraction is the process of audio-based music analysis. The general audio content analysis process includes signal preprocessing, audio feature extraction, and music content classification and inference. Audio signal preprocessing can reduce the total amount of processed data, eliminate irrelevant and interfering information, and enhance audio robustness. Audio feature extraction is the basis for all music content analysis, which analyses and extracts semantically rich information from the audio signal to obtain a compact, machine-processable feature representation. From technical analysis, low-level feature descriptions for music content include the following five categories: statistical, technical features extracted from audio data; timbral characteristics; tonal features, including the relationship between pitches in the signal; intensity-related features, such as loudness; and time-related features, such as rhythm and beat position.

*(2) Score Knowledge Extraction*. Score knowledge extraction is a notation-based process of music content analysis. It is based on formal and structured encoding. MIDI, MusicXML, and MEI are the three most common types of score encoding. Knowledge of musical scores is processed using musical feature analysis tools such as Symbolic, Humdrum toolkit, and music21, which are used to obtain musical notation feature data related to pitch, melody, chord intervals, rhythm, instrument configuration, and voice parts. Similar to the audio-based knowledge extraction process, the symbolic feature data and machine learning techniques can also be used for deep knowledge acquisition, such as musical style analysis and anonymous composer identity analysis.

*(3) Choral Knowledge Extraction*. Choral knowledge extraction can be referred to as a textual knowledge extraction process. This process also requires the use of natural language processing techniques. However, knowledge extraction of sung words needs to be supported by audio analysis techniques. The knowledge extraction tasks that can be accomplished using song lyrics as the object of knowledge acquisition include (1) singing structure analysis: the convolutional neural network is trained to accurately identify the repetitive structure in the self-similarity matrix encoding. It is also able to predict the position of the sung segments and mark different passages of the sung words at the corresponding positions in the audio. (2) Theme distribution detection: combining data training and manual annotation, a theme judgment model based on lyrics can be obtained. The theme model is then used to analyze the lyric data and obtain information on the theme distribution of the songs. (3) Lyrics summary extraction: based on the strong correlation between lyrics and audio, the audio scaling map technique was used to find representative fragments of the music. This is then combined with graphical and thematic analysis methods to form a summary of the lyrics. (4) Emotion description: by training an emotion recognition model, it is possible to determine the emotional tendencies expressed in the lyrics (positive or negative) and even to describe more explicit emotions.

#### 2.1.2. Musical Knowledge Integration

Knowledge fusion is a high-level knowledge organization that enables the integration of heterogeneous data from different knowledge sources under the exact framework specification. The steps to achieve this include ontology construction, entity alignment, entity linking, and ultimately the fusion of data, information, methods, experience, and ideas to form a high-quality knowledge graph.

*(1) Ontology Construction*. The music online education ontology build is the knowledge framework of the music knowledge graph. It is a critical step in the fusion of music knowledge, detailing the types of conceptual entities and the types of relationships between entities, setting the knowledge specification for the subsequent extraction process of education data. The ontology construction in this paper uses a manual construction approach.

The manual construction approach is combined with guidance from domain experts to artificially define constraints related to concept entity types, relationship types of concept entities, etc.  Figure 3 shows the top-level ontology of the manually constructed educational knowledge map. The subject knowledge ontology is a number of attributes corresponding to knowledge points, such as concepts and definitions. The curriculum standard ontology includes some teaching units including teaching objectives and teaching activities. The learning resources ontology covers teaching resources such as textbooks and microlessons.

*(2) Entity Alignment*. Entity alignment is taking entities from different data sources and corresponding them to the same entity to which they collectively refer. An essential task in knowledge fusion in the music domain is to complete the entity alignment of core entities such as musicians, musical works, and musical instruments.

String similarity-based entity alignment is where text or metadata in the form of cues associated with entities are analyzed for similarity. In most cases, the entity names and entity descriptions obtained by the music knowledge graph integration are ambiguous. There is no consistent representation form or identifier for the work names and artist information involved. Furthermore, multiple versions of musical works are prevalent, with different versions of the score, performance orchestration, performance venues, rips, transcriptions, etc., all producing different audio versions and corresponding titles in multiple languages and grammatical expressions. For this reason, it is tough to align musical works and musicians solely based on string similarity in the process of automatic entity alignment, which requires inference using all available information, followed by a review and correction process involving human intervention.

*(3) Physical Links*. While ontology construction and entity alignment complete the internal knowledge fusion of the knowledge graph, entity linking links disambiguated entities to external authoritative knowledge bases to achieve knowledge fusion between the knowledge graph and external data sources. dBpedia, as a cross-domain comprehensive knowledge base, plays a pivotal role in the interconnection of the knowledge graph. In the construction of music knowledge graphs, entities such as musicians, musical works, musical instruments, and musical concepts in dBpedia are often selected as entities to be linked. The LinkedBrainz knowledge graph is the preferred entity linking object for building the knowledge graph of music research because of the richness of music-related entities such as musical works, musicians, records, and singles. By linking to it, it can also be extended to retrieve the audio characterization data provided by AcousticBrainz, including pitch, rhythm, timbre, and other information.

#### 2.1.3. Music Knowledge Retrieval and Reasoning

In the Music Knowledge Graph, music knowledge retrieval can be achieved directly by constructing query statements using the SPARQL language. In addition, this can be achieved by natural language forms and example-based knowledge retrieval. Among them, relevance and similarity retrieval based on musical examples is a unique knowledge discovery approach in the music domain, which belongs to music content-based retrieval. This type of retrieval requires deep semantic processing of music content data by the knowledge graph. For audio data, audio feature extraction techniques are used to obtain content feature data, which is then organized and stored according to the audio analysis class ontology. For score-encoded data, an RDF transformation of the score using the score-related ontology is required. Through the profound fusion of musical knowledge of different representation types in the construction process, retrieval and discovery of examples and target entities across resource types can be achieved. For example, feature analysis of an audio paradigm can lead to discovering a target entity with the same or similar feature values, which can be audio or sheet music. Music knowledge inference is the inference of unique relationships between entities or new properties of entities within entity relationships.

### 2.2. Personalized Recommendation Methods for Online Music Education

A knowledge map of online music education with a fusion of multimodal resources can help learners choose more targeted learning resources and better learning styles. In teaching scenarios, many multimodal course resources are generated to help students understand relevant knowledge points. Still, the current course resources often stand alone and are not well connected to the knowledge points, failing to play the role of multimodal resources in interpreting the knowledge points. At the same time, the overall framework of course knowledge is mainly presented in the chapter table of contents in the book. In contrast, the relationships between the subtle knowledge points and knowledge points contained in the chapters are not very clear, making it difficult from the student's perspective to make connections between what has been learned before and after, and accepting knowledge remains difficult. Multimodal course knowledge mapping can effectively solve the above problems and assist in modeling course knowledge by mining a large number of course resources in authoritative textbooks and Internet platforms. In addition, the music knowledge map can integrate multimodal learning contents for learners and recommend relevant learning resources for them according to their learning progress, which can, to a certain extent, stimulate learners' enthusiasm and improve their learning efficiency. At the same time, using the rich semantic relationship representation between entities in the academic knowledge graph can help improve the problems of data sparsity and cold start in traditional recommendation algorithms and further enhance the quality of the recommendation system. Therefore, a personalized recommendation model for music online education courses is proposed (as illustrated in Figure 4).

#### 2.2.1. Graph Embedding

The graph embedding layer obtains embedding representations of relationships and entities at the triad level, learning item, and user representations with structural information at a fine granularity, improving the representation of users and items in the model and improving recommendation performance. In this paper, the TransR algorithm is used to learn embedding representations for multimodal knowledge graphs. The algorithm enables different entity types to be mapped into the same relational space by modeling entities and relations in different embedding spaces. Given the knowledge items (*h*, *r*, *t*) in the knowledge graph, the embedding representations *h*_*r*_ and *t*_*r*_ of the head and tail entities mapped from the relationship space are obtained by embedding representation learning.

(1) $$\begin{array}{c} h_{r}=hW_{r},\\ t_{r}=tW_{r}, \end{array}$$

where *W*_*r*_ is the transformation matrix for mapping from entity space to relationship space and the scoring function gr (*h*, *t*) calculates the deviation in the relationship space corresponding to the two entities.

(2) $$\begin{array}{c} g_{r}\left(h,t\right)=h_{r}+r-t_{r2}^{2}. \end{array}$$

The smaller the rating function gr (*h*, *t*) rating indicates, the greater probability that the triad is a fact. The algorithm is trained to take into account the relative order between positive and negative example triads, using a pairwise ranking loss function.

(3) $$\begin{array}{c} L_{1}=\sum_{\left(h,r,t,t\right)\in N}-\text{ln}\sigma \left(g_{r}\left(h,t\right)-g_{r}\left(h,\tilde{t}\right)\right), \end{array}$$

where $N=\left\{\left(h,r,t,\tilde{t}\right)\left(h,r,t\right)\in G,\left(h,r,\tilde{t}\right)\notin G\right\}$, *G* is the knowledge graph, the negative example triples are generated by random substitution, and *σ* (·) is the sigmoid activation function.

#### 2.2.2. Intralayer Propagation

The knowledge graph contains user entities, project entities, and related attributes of the project. The relationships between entities are rich in associative knowledge. Furthermore, neighboring entities are strongly correlated with each other, and layer-by-layer knowledge can be obtained through link propagation of the knowledge graph. As the level of propagation increases, different levels of entity sets and triples can be obtained, which contain higher-order associative knowledge and user interest. The valid information of different levels enriches the vector representation of users and items.

There are a large number of triad sets for each layer of users and projects, so the number of triads in each layer needs to be fixed. Users and projects are propagated in the same way in the graph, and this paper uses *o* as a placeholder; *o* can represent user *u* and project *v*. The head entity *h* in the high level triad set *B*_*o*_^*l*^ originates from the triad set *B*_*o*_^*l*−1^ in the previous layer and passes information through the intralayer propagation.

(4) $$\begin{array}{c} B_{o}^{l}=\left\{\left(h,r,t\right)|\left(h,r,t\right)\in G,h\in B_{o}^{l-1}\right\}, \end{array}$$

where *l* is the propagation level. For a user or item, the importance of entity nodes corresponding to different relationships is different, and therefore, the importance of neighbors needs to be distinguished during intralevel propagation. A scaling-aware attention mechanism can effectively distinguish the importance between neighboring entities in the propagation process at the same level, making the embedding representation of users and items more accurate.

Assume that the *i*-th triad representation of a user or item at layer *l* in the knowledge graph is (*h*, *r*, *t*). The tail entity node embedding representation *q*_*i*_ that joins the scaling-aware attention mechanism is derived from the product of the tail entity embedding representation *e*_*i*_^*t*^ and the attention weights.

(5) $$\begin{array}{c} q_{i}=f\left(e_{0}^{0},e_{i}^{h},r_{i}\right)e_{i}^{t}, \end{array}$$

where *e*_0_^0^ is the initial representation of the user. *e*_*i*_^*h*^ is the embedding representation of the head entity. *r*_*i*_ is the embedding representation of the relational entity. The attention network function *f* (·) calculates the attention weight of the tail entity *e*_*i*_^*t*^ which reflects the importance of the head entity to the tail entity nodes, and the scaling-aware attention function is defined as follows.

(6) $$\begin{array}{c} c_{0}=\text{ReLU}\left(M_{0}\left(e_{o}^{0}e_{i}^{h}r_{i}\right)+b_{0}\right),\\ f\left(e_{0}^{0},e_{i}^{h},r_{i}\right)=\sigma \left(M_{2}\text{ReLU}\left(M_{1}c_{0}+b_{1}\right)+b_{2}\right). \end{array}$$

The scaling-aware attention network splices together *e*_0_^0^, *e*_*i*_^*h*^ and *r*_*i*_ by a splicing operation, *M* and *b* are the parameters to be learned, different subscripts indicate different layers, and finally, the coefficients of the triplet are normalized using the SoftMax function. The attention network function *f* (·) is as follows:

(7) $$\begin{array}{c} f\left(e_{o}^{0},e_{i}^{h},r_{i}\right)=\frac{\exp\left(f\left(e_{o}^{0},e_{i}^{h},r_{i}\right)\right)}{\sum_{\left(h\prime ,r\right)\in B_{o}^{l}}\text{exp}{\left(f\left(e_{0}^{0},e_{i}^{h\prime },r_{i}\right)\right)}_{i}}. \end{array}$$

Aggregating the attentional embedding representations *q*_*i*_ of the tail entities in each layer of the triple yields the embedding representation *E*_*o*_^*l*^ of the user (item) at layer *l* of the propagation.

(8) $$\begin{array}{c} E_{o}^{l}=\sum_{i=1}^{\left|B_{a}^{l}\right|}q_{i}. \end{array}$$

*B*_*o*_^*l*^ is the total number of triples in layer *l*. The embedding of each layer represents an effective representation of the details of the propagation process, which can improve the expressiveness of the recommendation model.

#### 2.2.3. Interlayer Propagation

In the real world, user interest is not static. It may decay over time because they are tired of browsing too many similar items. Therefore, the model is not stable when propagating between multiple layers of user interest graphs. The interest information propagated needs to show a pattern of decay over time.

To simulate the propagation characteristics of user interest decaying, this paper designs a method for propagating interest based on a decay factor, where user interest exhibits an overall decaying characteristic when propagating between layers.

(9) $$\begin{array}{c} D_{u}^{L}=\mu_{1}E_{u}^{1}+\mu_{2}E_{u}^{2}+\cdots +\mu_{L}E_{u}^{L}, \end{array}$$

where *μ*_*i*_ and *D*_*u*_^*L*^ represents attenuation factor and interlayer user interest, respectively.

The knowledge graph recommendation method based on embedding propagation needs to pay attention to the problem of reduced semantic relevance during higher-order propagation when learning user and entity representations. To overcome this problem, this model uses user latent interest propagation in the higher-order propagation process to enhance the higher-order representation of users. Given the set of highest-order user triples *B*_*o*_^*L*^, a relevance probability *p*_*i*_ is assigned by comparing the items *v* of user interactions with the head entity *h* and the relationship entity *r*_*i*_ in each triple.

(10) $$\begin{array}{c} p_{i}=\text{softmax}\left(v^{T}r_{i}h\right)\\ =\frac{\exp\left(v^{T}r_{i}h\right)}{\sum_{\left(h,r,t\right)\in B_{o}^{L}}\text{exp}\left(v^{T}r_{i}h\right)}, \end{array}$$

where *r*_*i*_ and *h* can reflect the similarity between items and entities in the association space through relevance probabilities, in which the similarity between items and their corresponding entities varies across relationship conditions. The tailed entity *t* in the triplet with the corresponding relevance probability *p*_*i*_ weighted summation yields a higher-order representation of the user's potential interest *Z*_*u*_^*L*^, defined as follows:

(11) $$\begin{array}{c} Z_{u}^{L}=\sum_{\left(h,r_{i},t\right)\in B_{o}^{L}}p_{i}t. \end{array}$$

The end-user interest representation for interlayer propagation is a weighted average of the interlayer user interest representation *D*_*u*_^*L*^ and the higher-order potential interest representation *Z*_*u*_^*L*^:

(12) $$\begin{array}{c} T_{um}^{L}=\alpha D_{uw}^{L}+\beta Z_{u}^{L}, \end{array}$$

where *α* and *β* denote the weighting coefficients, and the values taken in this paper are *α* = 0.5 and *β* = 0.9.

#### 2.2.4. Enhanced Network-Based User Representation

Although the model has enhanced the representation of user interest for interlayer propagation, the algorithm's predictions using *T*_*u*_^*L*^ cannot yield good recommendations.

This is because the user interest representation suffers from data noise and degradation when the depth of the propagation layers and the depth of the propagation path is too large. To overcome this problem, this paper designs an augmented network with residual blocks to capture the focus of the current interest representation, reduce the noise caused by different paths, and thus improve the user interest representation.

As shown in Figure 5, the model takes two-by-two combinations of user interest representations as input parameters to the residual block and outputs enhanced user interest representations *H*_*u*_^1^, *H*_*u*_^2^, ⋯, *H*_*u*_^*k*^.

(13) $$\begin{array}{c} H_{u}^{k}=T_{u}^{k}+\delta \left(T_{u}^{k-1}\right), \end{array}$$

where *T*_*u*_^*L*^ is the directly mapped part of the residual block and *δ*(·) represents the residual network. Specially, set *H*_*u*_^1^ = *T*_*u*_^1^.

The model then stitches together the enhanced user interest representations and projects them to obtain the final user vector.

(14) $$\begin{array}{c} e_{u}=C\left(H_{u}^{1}H_{u}^{2}\ldots \left\|\right)H_{u}^{K}\right), \end{array}$$

where || denotes the splicing symbol and *C*(·) denotes the linear mapping function.

#### 2.2.5. Forecasting

*e*_*u*_ and *e*_*v*_ are the final representations of the user and the item, respectively. The inner product is used to predict the user-item preference score. The score size represents the probability of user interaction with the item.

(15) $$\begin{array}{c} {\hat{y}}_{uv}=e_{v}⊗e_{v}. \end{array}$$

For the optimization problem of the model, negative interactions were randomly selected from the user's unobserved interactions to ensure accurate experimental results. And, the sample sizes of positive and negative interactions were the same. The effectiveness of the model was evaluated using a cross-entropy loss function.

(16) $$\begin{array}{c} L_{2}=\sum_{u\in U}\left(\sum_{v\left(u,v\right)\in p^{+}}\pi \left(y_{uv},{\hat{y}}_{uv}\right)-\sum_{v\left(u,v\right)\in p^{-}}\pi \left(y_{uv},{\hat{y}}_{uv}\right)\right), \end{array}$$

where *π*(·) is the cross-entropy loss function. *p*^+^ indicates the positive user interactions. *p*− indicates negative user interactions. The final loss function of the model contains the loss of the knowledge graph embedding part and the recommendation part, i.e.,

(17) $$\begin{array}{c} L=\lambda_{1}L_{1}+\lambda_{2}L_{2}, \end{array}$$

where *λ*_*i*_ is the equilibrium hyperparameter, *λ*_1_ *=* *λ*_2_ = 0.5.

## 3. Result Analysis and Discussion

In this paper, experiments will be conducted on two mainstream datasets, Book-Crossing, a book dataset, and Last.FM, a music dataset, respectively [19]. These two datasets are both explicit feedback data. To better reflect the model recommendation performance, it needs to be converted to implicit feedback. Therefore, the dataset is randomly divided into training, validation, and test sets in the ratio of 6 : 2 : 2. The underlying statistics of the dataset are shown in Table 1.

### 3.1. Experimental Setup

The values of the main parameters of the proposed model are referred as the range of experimental parameters in the mainstream recommended models. The optimal parameter settings were finally derived by analyzing the relevant features of the dataset for experimentation in the experimental phase. The training set is batch processed. The learning rate is set to 1–4. The batch size is set to 128. The number of training rounds is set to 100. The increase in embedding vector dimension, hierarchical propagation depth, and the number of hierarchical triples brings exponential computational effort to the model. The recommended results do not increase much, and even exceeding a certain threshold brings the opposite result. Therefore, the embedding vector dimension *D is* chosen to be 64. The hierarchical propagation depth *L* is 4. And, the number of hierarchical triples is chosen to be 128. The model was optimized using the Adam optimizer. The model parameters were initialized using the Xavier initializer. The size of the augmented network on the book and music datasets was set to 8 and 12.

Due to the high correlation between entities and clicked items within a certain number of layers of the user interest graph, the interest of users is high. After a certain number of layers, the correlation between entities and clicked items decreases and user interest decays faster. The distribution of decay factors is not equivalent or satisfies exponential growth. The design method for the attenuation factors in the model uses a nonequivalence approach. It is assumed that user interest decays at different rates at each level of user interest and that the corresponding decay factors are independent. The attenuation factor is therefore set as a hyperparameter with initial values conforming to normal distribution.

To verify the effectiveness of the proposed model, *F*1 and AUC2 metrics were chosen to evaluate the model during the CTR click-through rate prediction task. Recall@K and Precision@K metrics were used in the Top-K recommendation task, where the values of *K* were 5, 10, 20, 50, and 100, respectively. Ten experiments were conducted for all experiments with random initialization. All experiments will be conducted 10 times with random initialization, and the mean value of the 10 experiments will be taken as the final experiment result.

### 3.2. Ablation Experiments

To investigate the effect of the augmented network size on the performance of the model, experiments were conducted on 2 datasets with different augmented network sizes *n.*Figure 6 gives the experimental results. The best results can be given to the model in which the *K* value is set to 8 and 12 on the book and music datasets, respectively. As the value of K increases, the performance of the model gradually rises. While the *K* value is above a threshold, the model performance decreases rapidly.

To verify the contribution of the intralayer interest propagation method based on the scaling-aware attention mechanism, the interlayer interest propagation method based on the fading factor, and the augmented network based on the residual blocks to the model, ablation experiments were conducted on 2 experimental data to demonstrate the advancement of the three. The experimental results are shown in Figures 7 and 8, where model 1 represents the model proposed in this paper. Model 2 represents model 1 with the intralayer interest propagation method based on the scaled attention mechanism removed. The embedding representation of the tail entity is directly aggregated to represent the embedding representation of this interesting mapping. Model 3 represents the removal of the interlayer interest propagation method based on fading factors and the direct aggregation of all interest graphs to represent the user interest graph representation. Model 4 indicates that the model removes the purification network with residual blocks and uses the interest graph representation obtained from the interlayer interest propagation method for recommendation prediction. The performance of the model with all three methods removed is significantly reduced compared to model 1, which demonstrates that the three methods do provide performance improvements to the model. Model 3 has the most significant performance drop due to the removal of the interlayer interest propagation method, followed by model 4, and the smallest drop due to the reduction of the intralayer interest propagation method in model 2.

### 3.3. Comparison Experiments

To further validate the performance metrics of the model, the experimental results of the proposed model are compared with other state-of-the-art models such as the Ripplenet model of literature [16], KGAT model of literature [17], KGCN model of literature [20], HKIPN model of literature [21], and PHGR model of literature [22].

The CTR prediction results of the present model on the two datasets obtained after several experiments are shown in Table 2. In the CTR prediction, the proposed model performs the best test results of AUC and *F*1 on the two sparse datasets, significantly better than the other comparable models. Compared to the state-of-the-art baseline model, the proposed model improved the AUC metrics by 3.36% and 2.49% on the Book-Crossing and Last.FM datasets, respectively, and the *F*1 metrics by 6.73% and 3.18%, respectively. Specifically, compared to the model of literature [20] and the AUC and *F*1 values of the model of literature [17] incorporating the attention mechanism, the model of literature [21] and this paper show significant improvements, indicating that the recommendation model incorporating the attention mechanism can more accurately learn the embedding representation of users and items during the dissemination process. The model of literature [16, 17, 20, 21] and the model proposed in this paper all use propagation for personalized recommendation. Cause of the model in literature [16] performs higher-order propagation representation learning unilaterally from the user's perspective. The advantage of the model in this paper is that it performs higher-order propagation representation learning from the perspective of user-project interactions on a collaborative knowledge graph. The models in literature [17] and literature [21] fuse user-item interaction information into the knowledge graph for obtaining higher-order information about users and items. The model in this paper builds on this by using user-item interaction information in interlayer propagation to further improve knowledge relevance in the higher-order propagation process.

In the Top-K recommendation task, all experiments are performed after the model has been trained to recommend the *K* items with the highest match for each user. Figures 9–12 present the Recall@K and Precision@K results for the Top-K recommendation task on the two datasets for different models. The proposed model achieves the best performance in the Top-K recommendation for the two datasets. Taking *K* = 20 as an example, the proposed model improved the Precision@20 metric by 7.6% and 16.91% on the Book-Crossing and Last.FM datasets, respectively. The Recall@20 metric by 7.6% and 16.91%, respectively, fully validated the effectiveness of the proposed algorithm in this paper.

## 4. Conclusion

In this paper, a multimodal music knowledge graph applicable to online music education in colleges and universities is constructed based on an indepth analysis of the characteristics of music knowledge graphs. To improve the learning efficiency of music online education, a personalized course recommendation method based on the embedded propagation knowledge graph is designed by mining the interest data of online education users. The proposed model analyses users' learning duration and ratings of courses, predicts users' preferences, and improves the accuracy of personalized course recommendations in online education systems by using user interest enhancement techniques. The experimental results on 2 datasets well validate the effectiveness of the model. The interaction between users and items in the model is still not tight enough. In the future, it is planned to combine user social networks into the model in this paper. The knowledge graph is integrated with user information to generate a heterogeneous information network containing user information and item information to better model the interaction between users and items. The structural-semantic information is explored to enhance the accuracy and interpretability of the recommendation system.

## Figures and Tables

**Figure 1:** Two ideas for the construction of multimodal knowledge graphs.

**Figure 2:** Framework diagram for building a music knowledge graph.

**Figure 3:** Top-level ontology for manually constructed knowledge graphs.

**Figure 4:** Personalized course recommendations with multimodal knowledge graphs.

**Figure 5:** Enhanced network with residual blocks.

**Figure 6:** Results of enhanced network scale experiments. (a) Book-Crossing. (b) Last.FM.

**Figure 7:** Ablation experiments on Book-Crossing.

**Figure 8:** Ablation experiments on Last.FM.

**Figure 9:** Recall@K experiment on Book-Crossing.

**Figure 10:** Recall@K experiment on the Last.FM.

**Figure 11:** Precision@K experiment on Book-Crossing.

**Figure 12:** Precision@K experiment on the Last.FM.

**Table 1:** Data set information.

Dataset		Book-Crossing	Last.FM

User-item interactions	Users	17860	1872
	Items	14967	3846
	Interactions	139746	42346

Knowledge graph	Triples	19793	15518
	Entities	77903	9366
	Relations	25	60

**Table 2:** Experimental results for CTR prediction.

Model	Book-Crossing		Last.FM	
	AUC	*F*1	AUC	*F*1

Proposed method	**0.768**	**0.729**	**0.866**	**0.778**
Literature [16]	0.721	0.647	0.778	0.702
Literature [17]	0.732	0.654	0.825	0.739
Literature [20]	0.684	0.631	0.802	0.722
Literature [21]	0.743	0.667	0.845	0.754
Literature [22]	0.736	0.683	0.819	0.75

## Data Availability

The labeled data set used to support the findings of this study is available from the corresponding author upon request.
